This article has been retracted.

# Resveratrol inhibits IL-1β-mediated nucleus pulposus cell apoptosis through regulating the PI3K/Akt pathway

**DOI:** 10.1042/BSR20190043

**Published:** 2019-03-26

**Authors:** Yanhai Jiang, Zhijie Xie, Jinying Yu, Lianqiang Fu

**Affiliations:** Department of Orthopaedics, The Affiliated Weihai Second Hospital of Qingdao University, Weihai 264200, China

**Keywords:** apoptosis, intervertebral disc degeneration, IL-1β, nucleus pulposus, resveratrol

## Abstract

Nucleus pulposus (NP) cell apoptosis is a classical cellular character during intervertebral disc degeneration (IDD). Previous studies have shown that inflammatory cytokine-induced NP cell apoptosis plays an important role in disc degeneration. The present study was aimed to investigate whether resveratrol can suppress IL-1β-mediated NP cell apoptosis and the potential signal transduction pathway. Experimental rat NP cells were treated with culture medium containing IL-1β (20 ng/ml) for 7 days. Control NP cells were cultured in the baseline medium. Resveratrol was added along with culture medium to investigate its effects. The inhibitor LY294002 was used to study the role of the PI3K/Akt pathway. NP cell apoptosis was reflected by the caspase-3 activity, cell apoptosis ratio, and expression of apoptosis-related molecules (Bcl-2, Bax, caspase-3, cleaved caspase-3, and cleaved PARP). Compared with the control NP cells, IL-1β significantly increased caspase-3 activity, NP cell apoptosis ratio and mRNA/protein expression of Bax, caspase-3, cleaved caspase-3 and cleaved PARP, but decreased mRNA expression of Bcl-2. However, resveratrol partly suppressed the effects of IL-1β on those cell apoptosis-related parameters. Further analysis showed that IL-1β significantly decreased activity of the PI3K/Akt pathway whereas resveratrol partly increased activity of the PI3K/Akt pathway in NP cells treated with IL-1β. Additionally, when the inhibitor LY294002 was added along with the resveratrol, its protective effects against IL-1β-induced NP cell apoptosis were attenuated. In conclusion, resveratrol suppresses IL-1β-mediated NP cell apoptosis through activating the PI3K/Akt pathway. Resveratrol may be an effective drug to attenuate inflammatory cytokine-induced disc degenerative changes.

## Introduction

With the aging of world population trends, many people suffer from low back pain, which causes a large medical cost to the health care system and seriously affects patient’s family economy [1,2]. Previous studies have confirmed that intervertebral disc degeneration (IDD) is an important contributor to low back pain [3]. Though lots of studies on pathogenesis and possible treatments of disc degeneration have been performed recently, there is still a long way to successfully retard disc degeneration.

Nucleus pulposus (NP) tissue is the central region of an intervertebral disc organ which contains a limited number of NP cells [4]. Normally, NP cells synthesize and secret extracellular matrix including aggrecan and collagen II to support the mechanical function of the disc [5]. Numerous studies have confirmed that NP cell apoptosis plays an important role during disc degeneration, which ultimately leads to the decrease in NP matrix synthesis [6–13]. In light of this point, inhibition of excessive apoptosis of NP cells may be an effective treatment to retard the progression of disc degeneration.

Currently, a consensus has been reached that disc degeneration is a process that is partly regulated by the inflammation response [14]. Lots of previous studies have investigated the effects of inflammatory cytokines on disc cell’s biology, such as cell apoptosis, cell senescence, and cellular metabolism [15–24]. Hence, inhibition of inflammation response-mediated cellular damage may be promising to retard disc degeneration.

Resveratrol, a natural phytoalexin found in plants [25], has a wide protective effects in different cell types, such as anti-inflammatory, anti-aging, and cartilage protection [26–28]. In recent several years, many researchers have demonstrated that resveratrol has protective effects against external pathological factors-induced degenerative changes in disc cells [11,20,29–41]. However, whether resveratrol can suppress inflammatory cytokine-induced NP cell apoptosis remains unclear. In the present study, we mainly aimed to study the effects of resveratrol on apoptosis of NP cells treated with IL-1β.

## Materials and methods

### NP cell isolation and culture

All animal procedures were approved and performed according to the guidelines of the Ethics Committee of Qingdao University (SHNK[E] 2011-021). Lumbar spinal columns were separated from male or female Sprague–Dawley rats (400 g, 12-weeks old) under aseptic conditions. After the central NP tissues were separated under a dissecting microscope, they were sequentially incubated with 0.25% trypsin for 5 min and 0.2% type I collagenase for 15 min at 37°C. Then, the cell pellets were transferred to a culture bottle containing DMEM/F12 medium supplemented with 15% fetal bovine serum (FBS, Gibco, U.S.A.). When reaching confluence (after approximately 8 days), NP cells were dissociated using 0.25% trypsin and sub-cultured. The passage 3 NP cells were used for each experiment in the present study. IL-1β (20 ng/ml) was added into the culture medium to induce NP cell apoptosis for 7 days in the experiment group, as described by a previous study [22]. NP cells treated with nothing were regarded as control cells. Resveratrol (100 μM) was added along with the culture medium in the experiment group to investigate its effects [40]. The inhibitor LY294002 (10 μM) was used to further investigate the role of the PI3K/Akt pathway in this process.

### Flow cytometry assay

NP cell apoptosis was measured using a Annexin V-FITC Apoptosis Detection Kit (Beyotime, China). Briefly, after NP cells were incubated with the test compounds for 7 days, they were washed with sterile PBS for three times. Then, they were dissociated by 0.25% trypsin without EDTA and incubated with test solution in the chemical kit according to the manufacturer’s instructions. Finally, apoptotic NP cells were analyzed by FACS scan flow cytometer (ACEA Biosciences, U.S.A.).

### Caspase-3 activity measurement

Caspase-3 activity was studied using a Caspase-3 Activity Assay Kit (Beyotime, China). Briefly, after NP cells were incubated for 7 days with different test compounds, they were washed with PBS for three times. After they were lysed using the lysis buffer in the kit, protein concentration was determined using a BCA Protein Assay Kit (Beyotime, China). Then, a standard curve was created using the standard provided by the chemical kit. Finally, the reaction system was used to measure the absorbance value at a wavelength of 405 nm to calculate caspase-3 activity.

### RNA extraction and real-time PCR

Briefly, after NP cells were incubated for 7 days with different test compounds, the total RNA was extracted using a RNeasy Mini Kit (Qiagen Inc., Valencia, CA). Then, the contaminating DNA was removed, and RNA was reverse-synthesized into cDNA using a Transcriptor First Strand cDNA Synthesis Kit (Roche, Indianapolis, IN). Finally, real-time PCR was performed using the SYBR Green PCR Master Mix (Applied Biosystems, CA, U.S.A.) to detect the mRNA expression of caspase 3, Bax, and Bcl-2. PCR reactions were: 3 min at 95°C, followed by 40 cycles of 30 s at 95°C, 25 s at 58°C, and 15 s at 72°C. The gene primers were presented in the Table 1. The relative gene expression was normalized to GAPDH and calculated with the method of 2^−ΔΔC^_t_.

**Table 1:** Primers of target genes

Gene	Forward (5’-3’)	Reverse (5’-3’)
GAPDH	GTATTGGGCGCCTGGTCACC	CGCTCCTGGAAGATGGTGATGG
Bcl-2	ATGTGTGTGGAGAGCGTCAA	ACAGTTCCACAAAGGCATCC
Bax	GGGGACGAACTGGACAGTAA	TTGAAGTTGCCGTCAGAAAA
Caspase 3	CTGGACTGCGGTATTGAGAC	CCGGGTGCGGTAGAGTAAGC

### Protein extract and Western blot assay

After being cultured for 7 days in different test compounds, they were washed with PBS for three times. Then, they were lysed by Cell Lysis Buffer for Western and IP (Beyotime, China) according to the manufacturer’s instructions, followed by protein concentration analysis using a BCA Protein Assay Kit (Beyotime, China) and denatured in SDS–PAGE Sample Loading Buffer at 100°C for 5 min. Then, the protein samples were transferred onto the PVDF membrane and incubated with the primary antibodies (β-actin: Cell Signaling Technology, #3700; cleaved caspase-3: Cell Signaling Technology, #9644; cleaved PARP:Cell Signaling Technology, #94885; Akt: Cell Signaling Technology, #4691; p-Akt: Cell Signaling Technology, #4060) and secondary antibodies according to the standard Western blot experiment procedures. After protein bands were detected by the enhanced ECL reagent (Beyotime, China), the gray value of the protein bands was analyzed using the Image J software (Bethesda, MD, U.S.A.).

### Statistical analysis

All numeric data in the present study were expressed as mean ± standard deviation (SD) for three independent experiments. SPSS software (Version 19.0, U.S.A.) was used for statistical analyses. Statistical difference was analyzed using one-way analysis of variance (ANOVA). A p value of less than 0.05 was considered as a statistically significance.

## Results

### NP cell apoptosis ratio

To evaluate NP cell apoptosis, cell apoptosis ratio was first analyzed by flow cytometry. Results showed that IL-1β significantly increased cell apoptosis ratio compared with the control NP cells. Resveratrol partly decreased cell apoptosis ratio in IL-1β-treated NP cells. Additionally, the inhibitor LY294002 partly increased cell apoptosis ratio in NP cells treated with the mixture containing both IL-1β and resveratrol (Figure 1).

**Figure 1:** Analysis of cell apoptosis ratio of NP cells Data are expressed as mean ± SD, *n*=3. *: Significant difference (*P*<0.05) between two groups. Abbreviations: LY, LY294002; Res, resveratrol.

### Caspase-3 activity

Caspase-3 activity is a common parameter to reflect cellular apoptosis. Here, its activity was measured using a chemical kit. Results showed that IL-1β obviously increased caspase-3 activity compared with the control NP cells. Resveratrol partly decreased caspase-3 activity in IL-1β-treated NP cells. The inhibitor LY294002 partly increased caspase-3 activity in NP cells treated with IL-1β and resveratrol (Figure 2).

**Figure 2:** Analysis of caspase-3 activity in NP cells Data are expressed as mean ± SD, *n*=3. *: Significant difference (*P*<0.05) between two groups. Abbreviations: LY, LY294002; Res, resveratrol.

### Gene expression analysis of apoptosis-related molecules

Gene expression of anti-apoptosis molecule (Bl-2) and pro-apoptosis molecules (Bax and caspase-3) was analyzed here. We found that IL-1β significantly up-regulated expression of Bax and caspase-3, and down-regulated expression of Bcl-2. However, their expression profile was partly reversed by addition of resveratrol in NP cells treated with IL-1β. When the inhibitor LY294002 was added into the culture medium of NP cells treated with IL-1β and resveratrol, their expression profiles partly showed an opposite trend (Figure 3).

**Figure 3:** Gene expression of apoptosis-related molecules in NP cells Data are expressed as mean ± SD, *n*=3. *: Significant difference (*P*<0.05) between two groups. Abbreviations: LY, LY294002; Res, resveratrol.

### Protein expression of apoptosis markers

Cleaved caspase-3 and cleaved PARP are two important parameters which directly indicate the cellular apoptosis process. To investigate the changes of NP cell apoptosis among those groups, protein expression of apoptosis markers (cleaved caspase-3 and cleaved PARP) was analyzed. Results showed that IL-1β increased protein expression of cleaved caspase-3 and cleaved PARP, whereas resveratrol decreased protein expression of cleaved caspase-3 and cleaved PARP in NP cells treated with IL-1β. In addition, the inhibitor LY294002 partly increased their protein expression in NP cells treated with IL-1β and resveratrol (Figure 4).

**Figure 4:** Protein expression of apoptosis-related markers in NP cells Data are expressed as mean ± SD, *n*=3. *: Significant difference (*P*<0.05) between two groups. Abbreviations: LY, LY294002; Res, resveratrol.

### Analysis on the activation of the PI3K/Akt pathway

Activity of the PI3K/Akt pathway was expressed as the ratio of p-Akt protein expression to Akt protein expression. Results showed that IL-1β obviously decreased activity of the PI3K/Akt pathway compared with the control NP cells. However, addition of resveratrol partly increased activity of the PI3K/Akt pathway in IL-1β-treated NP cells. Predictably, the inhibitor LY294002 obviously decreased activity of the PI3K/Akt pathway in NP cells treated with IL-1β and resveratrol (Figure 5).

**Figure 5:** Analysis of activity of the PI3K/Akt pathway by Western blot assay Data are expressed as mean ± SD, *n*=3. *: Significant difference (*P*<0.05) between two groups. Abbreviations: LY, LY294002; Res, resveratrol.

## Discussion

Disc degeneration is an important risk factor of low back pain worldwide [42]. Until now, its pathogenesis is not fully understood though some mechanisms driving disc degeneration have been clarified. Among those mechanisms, disc cell apoptosis and inflammation response are proved to be closely related with disc degeneration [6–8,10,11,14–16]. Moreover, several studies have showed that inflammation response is directly related with disc cell apoptosis [20–22]. Hence, inhibition of inflammation response-induced NP cell apoptosis may be helpful to retard disc degeneration. As a phytoalexin identified in peanuts, grapes and other plants, resveratrol is found to have protective effects against inflammation response [43]. However, whether resveratrol can attenuate inflammation response-mediated NP cell apoptosis remains unclear.

In the present study, we investigated for the first time the effects of resveratrol on NP cell apoptosis in an inflammation environment. Compared with the control NP cells in the present study, we found that inflammatory cytokine IL-1β significantly increased cell apoptosis ratio, caspase-3 activity, up-regulated gene/protein expression of Bax, caspase-3, cleaved caspase-3 and cleaved PARP, and down-regulated gene expression of Bcl-2. These results indicate that IL-1β promotes NP cell apoptosis *in vitro*, which confirms previous studies demonstrating that inflammatory cytokines induce NP cell apoptosis [20–22]. However, we found that resveratrol supplementation partly decreased cell apoptosis ratio and caspase-3 activity, down-regulated gene/protein expression of Bax, caspase-3, cleaved caspase-3 and cleaved PARP, and up-regulated expression of Bcl-2 in NP cells treated with IL-1β. These results indicate that resveratrol attenuates inflammatory cytokine IL-1β-mediated NP cell apoptosis. These effects are in line with previous reports indicating the anti-inflammation effects of resveratrol [43]. Importantly, this is similar to the previous studies showing that resveratrol suppresses NP cell apoptosis induced by other pathological factors [11,33,41].

PI3K/Akt pathway mediates lots of cellular biological activities, such as cell proliferation, cell senescence, and cell apoptosis [44]. To investigate whether the PI3K/Akt pathway participates in this process, we evaluated its activity using Western blot assay. Results showed that IL-1β significantly inhibited activation of the PI3K/Akt pathway whereas resveratrol partly promoted activation of this pathway. In light of the opposite trend of parameters reflecting NP cell apoptosis among the control group, IL-1β group and IL-1β + resveratrol group, we deduced that PI3K/Akt pathway may be involved in the protective effects of resveratrol against IL-1β-induced NP cells apoptosis. Additionally, when the PI3K/Akt pathway was inhibited by the inhibitor LY294002, the protective effects of resveratrol against IL-1β-induced NP cell apoptosis were attenuated. This further indicates that resveratrol suppresses inflammation response-induced NP cell apoptosis through regulating the PI3K/Akt pathway.

In a word, the present study investigated the effects of resveratrol on IL-1β-induced NP cells apoptosis and the potential signaling transduction pathway. Our results again confirmed that inflammatory cytokine IL-1β significantly promoted NP cell apoptosis, and demonstrated that RSV partly suppressed IL-1β-induced NP cells apoptosis through activating the PI3K/Akt pathway. The present study helps us further understand the protective effects of resveratrol and indicates that resveratrol may be efficient in attenuating inflammation response-induced disc degeneration.

## Abbreviations

Bax: Bcl-2 assaciated X protein
Bcl-2: B-cell lymphoma-2
IDD: intervertebral disc degeneration
IL: interleukin
NP: nucleus pulposus
PI3K: phosphatidylinositol 3-kinase
RSV: resveratrol
